The article "Erchen Decoction Ameliorates the Metabolic Abnormalities of High-Fat Diet-Fed Rats" was retracted in 2023. Reasons: signs of a paper mill; suspected computer-generated content; unreliable results or conclusions; concerns about the data.

# Erchen Decoction Ameliorates the Metabolic Abnormalities of High-Fat Diet-Fed Rats

**DOI:** 10.1155/2022/2183542

**Published:** 2022-07-06

**Authors:** Ya Cheng, Lu-Yao Xu, Ning Zhang, Jun-Hua Yang, Li Guan, Hai-Mei Liu, Ya-Xing Zhang, Run-Mei Li, Jin-Wen Xu

**Affiliations:** ^1^The Research Center of Basic Integrative Medicine, Basic Medical College, Guangzhou University of Chinese Medicine, University Town, Guangzhou 510006, China; ^2^Department of Physiology, Basic Medical College, Guangzhou University of Chinese Medicine, University Town, Guangzhou 510006, China

## Abstract

**Objective:**

Brown adipose tissue (BAT) dissipates chemical energy to protect against obesity. In the present study, we aimed to determine the effects of Erchen decoction on the lipolysis and thermogenesis function of BAT in high-fat diet-fed rats.

**Methods:**

Sprague-Dawley rats were randomly divided into four groups, which were fed a control diet (C) or a high-fat diet (HF), and the latter was administered with high and low doses of Erchen decoction by gavage once a day, for 12 weeks. Body weight, the serum lipid profile, serum glucose, and insulin levels of the rats were evaluated. In addition, the phosphorylation and protein and mRNA expression of AMP-activated protein kinase (AMPK), adipose triglyceride lipase (ATGL), peroxisome proliferator-activated receptor *γ* coactivator- (PGC-) 1*α*, and uncoupling protein 1 (UCP-1) in BAT were measured by immunoblotting and RT-PCR.

**Results:**

Erchen decoction administration decreased body weight gain and ameliorated the abnormal lipid profile and insulin resistance index of the high-fat diet-fed rats. In addition, the expression of p-AMPK and ATGL in the *BAT* was significantly increased by Erchen decoction. Erchen decoction also increased the protein and mRNA expression of PGC-1*α* and UCP-1 in BAT.

**Conclusion:**

Erchen decoction ameliorates the metabolic abnormalities of high-fat diet-fed rats, at least in part *via* activation of lipolysis and thermogenesis in BAT.

## 1. Introduction

The prevalence of obesity has reached epidemic proportions, and 600 million people worldwide are estimated to be obese by 2025 [1]. The prevalence of obesity in China has risen rapidly in the past four decades [2]. Obesity is associated with unemployment, social disadvantages, and reduced socioeconomic productivity, thus increasingly creating an economic burden [3]. Furthermore, obesity has been shown to play an important role in the pathophysiology of numerous chronic diseases which include cardiovascular disease (CVD), dyslipidemias, type 2 diabetes (T2D), and cancer [4–6]. The fifth risk for attributable deaths in females was high body mass index (hBMI), while for the males, hBMI accounts for the sixth risk attributed to death in 2019 [7]. Although tremendous progress over the last decade has been made in treating obesity, the development of additional classes of therapeutics and drugs is still needed to be explored to reduce its burden.

Obesity develops when the metabolic energy input of the body exceeds the energy output. Human beings have two kinds of adipose tissue. White adipose tissue (WAT) stores the excess energy tissue in the form of triglycerides in a fat-storing droplet. In addition to WAT, mammals possess brown adipose tissue (BAT), which plays a nearly opposite function [8]. BAT has multilocular lipid droplets and large numbers of mitochondria that contain uncoupling protein-1 (UCP1). UCP-1 in BAT uncouples the respiratory chain from oxidative phosphorylation. This process allows brown adipocytes to actively oxidize substrates to produce heat [8]. Numerous studies reported that BAT-mediated thermogenesis can protect against obesity by promoting energy expenditure [9–11]. Thus, activation of the thermogenesis function of BAT is an expected way to treat obesity.

Erchen decoction (ECD) is a common prescription in traditional Chinese medicine (TCM) to treat obesity and its related diseases [12, 13]. ECD is composed of Pinellia ternata, tangerine peel, Poria cocos, and Glycyrrhiza uralensis. In the theory of TCM, Pinellia ternate and tangerine peel which are the main component of ECD are able to raise the PI function through activating lipid oxidation function of the skeletal muscle [14, 15]. It is reported that classical BAT in the interscapular depots and skeletal muscles are both derived from a myf-5 positive progenitor cell [16, 17]. Therefore, this study mainly investigates whether ECD could activate lipolysis and thermogenesis in BAT.

## 2. Methods

### 2.1. Animals

All the experimental procedures were performed in accordance with the Guidelines for Animal Experiments of the Committee of Medical Ethics of Guangzhou University of Chinese Medicine, National Health Department of China. Male Sprague-Dawley rats (220–250 g) were obtained from the Laboratory Animal Center at Guangzhou University of Chinese Medicine. The rats were randomly allocated to four groups, which were fed a control diet and orally administered physiological saline (CON group; *n* = 10), fed a high-fat diet (60% hydrogenated coconut oil; D12492; Research Diets, Inc; New Brunswick, NJ, USA) and orally administered physiological saline (HF group; *n* = 10), or fed high-fat diet and orally administered high and low doses of Erchen decoction (4.3 g/kg and 17.2 g/kg, once a day; ECDL and ECDH, *n* = 10) for 12 weeks.

### 2.2. Preparation of ECD and LC-MS/MS Analyses

The herbal components of ECD (Pinellia ternata, tangerine peel, Poria cocos, and Glycyrrhiza uralensis at a weight ratio of 3 : 3 : 2 : 1) were acquired from Kangmei Pharmaceutical Co., Ltd. (Guangzhou, China). The liquid extract obtained was concentrated at 0.435 g/mL and 1.74 g/mL under reduced pressure. ECD was stored under 4°C and reprepared once a week. The quality control for ECD concentrated granules has been evaluated by LC-MS/MS determined by Agilent 1290uplc and qtof6550 with a WATERS BEH C18 column (2.1∗100 mm 1.7 *μ*m). The injection volume was 5 *μ*L. The electrospray ionization source was set to positive and negative modes.

### 2.3. Tissue Collection and Biochemical Analysis

The rats were fasted overnight, and trunk blood was then obtained, left at room temperature for 30 min, and then centrifuged at 4,500 × *g* and 4°C for 15 min. The lipid concentrations and glucose levels of the serum obtained were measured using a Hitachi clinical analyzer. The plasma level of insulin was determined using Rat ELISA kits (Invitrogen Inc). To evaluate the degree of insulin resistance, the homeostasis model assessment (HOMA) was used as an index of IR and calculated by the following formula: insulin (mU/mL)∗glucose (mmol/L)/22.5 [18].

### 2.4. Histological Analysis

Tissue sections (5 mm) were obtained from epididymal visceral adipose and interscapular BAT samples that had been fixed and embedded in paraffin. These were then deparaffinized in xylene, rehydrated, and washed in phosphate-buffered saline, prior to hematoxylin and eosin (HE) staining. For immunohistochemical staining, endogenous peroxidase activity was quenched in hydrogen peroxide for 10–15 min, and the sections were washed four times in PBS buffer. Sections were then incubated with the primary antibodies, at 4°C overnight. And immunostaining was identified using DAB peroxidase substrate solution as the chromogen.

### 2.5. Real-Time Reverse Transcription-PCR

Real-time PCR was performed as previously described [19]. cDNA was synthesized using a Transcriptor First Strand cDNA Synthesis Kit (Roche, Basel, Switzerland), according to the manufacturer's instructions. For PGC1-*α*, the primers were 5′-CAACAATGAGCCTGCGAACA-3′ (forward) and 5′-TGAGGACCGCTAGCAAGTTTG-3′ (reverse), resulting in a 71 bp RT-PCR product. For UCP-1, the primers were 5′-GTGAAGGTCAGAATGCAAGC-3′ (forward) and 5′-AGGGCCCCCTTCATGAGGTC-3′ (reverse), resulting in a 100 bp RT-PCR product. For GAPDH, the primers were 5′-AGACAGCCGCATCTTCTTGT-3′ (forward) and 5′-CTTGCCGTGGGTAGAGTCAT-3′ (reverse), resulting in a 207 bp RT-PCR product. RT-PCR reactions were performed using a CFX96™ Real-Time System (Bio-Rad, Hercules, CA, USA) in final volumes of 20 *μ*L, which contained 10 *μ*L of FastStart Universal SYBR Green Master (Rox) (Roche, Basel, Switzerland), 1 *μ*L of each primer (10 *μ*M), 2 *μ*L of cDNA, and 7 *μ*L of PCR-grade water. The RT-PCR products underwent melting point analysis and were quantified using the *ΔΔ*CT method, with GAPDH as the reference gene. The expression in the HF and HF+CL groups was normalized to that of the C group.

### 2.6. Immunoblotting

Immunoblotting was performed as previously described [20]. Briefly, tissue lysates were separated by sodium dodecyl sulfate-polyacrylamide gel electrophoresis and then electrotransferred to membranes. The primary antibodies used were as follows: anti-UCP-1, anti-PGC-1*α* (PA5-22958; Thermo), anti-AMPK (5831; Cell Signaling Technology), anti-p-AMPK (2535; Cell Signaling Technology), anti-ATGL (2439; Cell Signaling Technology), anti-p-ATGL (135093; Abcam), and anti-glyceraldehyde 3-phosphate dehydrogenase (GAPDH) (5174; Cell Signaling Technology). Membranes were incubated with primary and secondary antibodies using standard techniques, and the detection of specific protein bands was accomplished using enhanced chemiluminescence. Images of the bands were acquired and analyzed using a quantitative digital imaging system (Quantity One; Bio-Rad), avoiding saturation.

### 2.7. Statistical Analysis

Data are presented as the mean ± standard deviation (SD) and represent the results of at least three independent experiments. Statistical comparisons were made using Student's *t*-test or one-way analysis of variance, followed by Tukey's test where applicable, to identify significant differences between mean values. *p* < 0.05 was considered to represent statistical significance.

## 3. Results

### 3.1. LC-MS/MS Analyses of ECD

The total ion chromatogram of ECD is shown in Figure 1. This was matched with the OTCML database. A total of 119 compounds in ECD were identified through chromatogram matching (Supplementary material 1). The concentration of hesperidin in ECD was 91.48 ppm.

### 3.2. ECD Administration Reduces the Body Mass and Ameliorates the Serum Lipid Abnormalities and Insulin Resistance of High-Fat Diet-Fed Rats

As expected, the body masses of the HF rats were significantly higher than those of the CON rats, but ECD administration reduced the body mass of the HF rats (Figure 2(a)). The HF rats had significantly higher total serum cholesterol, triglyceride, and low-density lipoprotein- (LDL-) cholesterol concentrations than the CON group, whereas the high-density lipoprotein- (HDL-) cholesterol concentration in the HF rats was significantly lower. However, ECD administration improved the lipid profile of the HF rats (Figure 2(b)). The HF rats had significantly higher serum glucose, and insulin levels and ECD administration reduced serum glucose and insulin levels (Figures 2(c) and 2(d)). Consistently, ECD administration reduced HOMA-IR in HF rats (Figure 2(e)).

### 3.3. ECD Administration Reduces the Epididymal Fat Depot Masses of HFD-Fed Rats

HE staining of tissue sections showed that HF rats had larger lipid droplets in their interscapular brown and epididymal adipocytes (Figure 3(a)). Concurrent ECD administration reduced the weight of epididymal adipose tissue fed with high-fat diet (Figure 3(b)).

### 3.4. ECD Administration Increases the Expression of UCP-1 and PGC-1*α* in the Interscapular Brown Adipose Tissue of HF Rats

ECD administration increased UCP-1 and PGC-1*α* mRNA expression in the interscapular BAT of HF rats (Figure 4(a)). Consistent with this, immunoblotting and immunohistochemistry assay showed that the protein expression levels of UCP-1 and PGC-1*α* in the interscapular BAT of HF rats were significantly lower than those of CON rats, and ECD administration eliminated these differences (Figures 4(b) and 4(c)).

### 3.5. ECD Treatment Increases p-AMPK and p-ATGL Expression in the Interscapular Brown Adipose Tissue of HF Rats

Immunoblotting showed that the protein expression levels of p-AMPK and p-ATGL in their interscapular brown adipose tissue of HF rats were significantly lower than those of CON rats, and ECD administration eliminated these differences (Figures 5(a) and 5(b)).

## 4. Discussion

Obesity is one of the most common metabolic diseases around the world partially due to the consumption of fast food containing high levels of fat and glucose [21, 22]. In the present study, we first found that high-fat diet for 12 weeks increased body weight and serum lipid profiles and exacerbated glucose tolerance and insulin sensitivity. In the theory of TCM, high-fat diet leads to Pi deficiency and increased dampness in the body. We also found that the epididymal visceral adipose tissue had larger lipid droplets which is a sign of increased dampness in the body after high-fat diet feed. ECD is clinically used in China to treat obesity and hyperlipidemia by its dampness-reducing effects [12, 13]. ECD has been also demonstrated to prevent high-fat diet-induced metabolic disorders [23–25]. Herein, we consistently found that ECD treatment was able to reduce body weight and serum lipid profiles in high-fat diet-fed rats. ECD treatment also significantly reduced the epididymal visceral adipose tissue weight and the diameter of the lipid droplets in the epididymal visceral adipose tissue. These results indicated that ECD was able to remove the phlegm in the form of triglyceride in adipose tissue.

It was previously thought that BAT was regressed in adulthood [26]. However, a large quantity of bioactive brown/beige adipocytes was recently found in the neck and shoulder regions of adults by 18F-FDG-PET/CT detection [27, 28]. This has sparked a resurgence in the targeting of BAT to treat obesity and type 2 diabetes. Many traditional Chinese medicine drugs have been shown to activate BAT to prevent metabolic disorders in high-fat diet-fed mice and rats [29–31]. According to the theory of TCM, high-fat diet-induced Pi deficiency leads to skeletal muscle dysfunction, while ECD increases Pi and has beneficial metabolic effects on high-fat diet-fed mice partially due to the upregulation of the protein levels of lipoprotein lipase in skeletal muscle. BAT and skeletal muscle both originated from myogenic factor 5 positive cells [16, 17]. Thus, we hypothesized that ECD might activate the thermogenesis function of BAT and found ECD was able to increase the protein and mRNA levels of UCP-1 in BAT. Peroxisome proliferator-activated receptor gamma coactivator 1 alpha (PGC-1*α*) serves as a master regulator for mitochondrial biogenesis and function, and it is highly expressed in BAT upon exposure of mice to cold [32]. PGC-1 plays a central role in thermogenesis through the upregulation of UCP-1 in BAT [33, 34]. Next, we consistently found that ECD also upregulated the protein and mRNA levels of PGC-1*α* in BAT in high-fat diet-fed rats.

Lipolysis is a fundamental biochemical process which occurs essentially in WAT and BAT. The catabolism of triglyceride molecules is through the activation of the major TAG hydrolases, such as adipose triglyceride lipase (ATGL) and hormone-sensitive lipase (HSL) [35]. Lipolytic activity of ATGL affects BAT function, and adipocyte-specific ATGL knockout (KO) mice show impaired thermogenic functions in response [36]. Furthermore, activation of AGTL in BAT was found to improve metabolic parameters in high-fat diet-fed mice [37]. Thus, we next detected the expression levels of p-ATGL in BAT and found that ECD was able to activate AGTL in BAT in high-fat diet-fed rats. AMP-activated protein kinase (AMPK) is a widely expressed multisubstrate serine/threonine kinase and a well-known sensor of the intracellular energy state that responds to metabolic stresses and other regulatory signals [38]. By sensing the cellular energy state, AMPK activation induces FA oxidation partially by phosphorylating ATGL to increase its TAG hydrolase activity [39]. Our results showed that ECD upregulated the expression levels of p-AMPK in BAT in high-fat diet-fed rats. These indicated that ECD might activate lipolysis in BAT partially through the AMPK-ATGL pathway.

## 5. Conclusions

In conclusion, the present study demonstrated that Erchen decoction improves metabolic parameters of high-fat diet-fed rats via activating lipolysis and thermogenesis in brown adipose tissue.

## Figures and Tables

**Figure 1:** Total ion current chromatogram of LC-MS/MS of ECD.

**Figure 2:** ECD treatment reduced the body weight and improved serum lipid profile and glucose tolerance in HFD-fed rats. Body weight (a), serum lipid profiles (b), serum glucose levels (c), serum insulin levels (d), and HOMA-IR of rats after treatment with ECD. AUC: area under the curve; ECD: Erchen decoction; CON: control group; HF: high-fat diet group; ECDL: high-fat diet and low dose of ECD treatment group; ECDH: high-fat diet and high dose of ECD treatment group. ^∗^*p* < 0.05 versus CON; ^#^*p* < 0.05 versus HF. Bars represent SD, *n* = 8.

**Figure 3:** ECD treatment reduced the weights of visceral periepididymal adipose tissue in HFD-fed rats. (a) Representative HE staining of visceral periepididymal adipose tissue and interscapular brown adipose tissue. Bar scale 200 *μ*m. (b) The weight of visceral periepididymal adipose tissue and interscapular brown adipose tissue. VAT: visceral periepididymal adipose tissue; BAT: interscapular brown adipose tissue; ECD: Erchen decoction; CON: control group; HF: high-fat diet group; ECDL: high-fat diet and low dose of ECD treatment group; ECDH: high-fat diet and high dose of ECD treatment group. ^∗^*p* < 0.05 versus CON; ^#^*p* < 0.05 versus HF. Bars represent SD, *n* = 8.

**Figure 4:** ECD increased the expression levels of UCP-1 and PGC-1*α* in interscapular brown adipose tissue in HFD-fed rats. (a) ECD increased UCP-1 and PGC-1*α* mRNA expression levels in interscapular brown adipose tissue in HFD-fed rats. UCP-1/GAPDH mRNA and PGC-1*α*/GAPDH mRNA levels were measured by qPCR. Expression in the CON group was normalized to 1, *n* = 4. (b) Representative immunohistochemical analysis showing the expression of UCP-1 in interscapular brown adipose tissue cross-sections. Bar scale 200 *μ*m. (c) ECD increased UCP-1 and PGC-1*α* protein expression levels in interscapular brown adipose tissue in HFD-fed rats. UCP-1 and PGC-1*α* densitometry values were adjusted to GAPDH intensity, then normalized to expression from the control sample. Expression in the CON group was normalized to 1, *n* = 3. ECD: Erchen decoction; CON: control group; HF: high-fat diet group; ECDL: high-fat diet and low dose of ECD treatment group; ECDH: high-fat diet and high dose of ECD treatment group. ^∗^*p* < 0.05 versus CON; ^#^*p* < 0.05 versus HF.

**Figure 5:** ECD activated AMPK/ATGL signaling. (a) ECD increased p-AMPK protein expression levels in interscapular brown adipose tissue in HFD-fed rats. p-AMPK densitometry values were adjusted to AMPK intensity, then normalized to expression from the control sample. Expression in the CON group was normalized to 1, *n* = 3. (b) ECD increased p-ATGL protein expression levels in interscapular brown adipose tissue in HFD-fed rats. p-ATGL densitometry values were adjusted to ATGL intensity, then normalized to expression from the control sample. Expression in the CON group was normalized to 1, *n* = 3. ECD: Erchen decoction; CON: control group; HF: high-fat diet group; ECDL: high-fat diet and low dose of ECD treatment group; ECDH: high-fat diet and high dose of ECD treatment group. ^∗^*p* < 0.05 versus CON; ^#^*p* < 0.05 versus HF.

## Data Availability

The datasets used and/or analyzed during the current study are available from the corresponding authors on reasonable request.

## Supplementary Materials

Supplementary Materials Supplementary material 1: a total of 119 compounds in ECD were identified through chromatogram matching.
